The article "Context-dependent interpretation of the prognostic value of BRAF and KRAS mutations in colorectal cancer" was published in 2013. Journal: BMC Cancer.

# Context-dependent interpretation of the prognostic value of BRAF and KRAS mutations in colorectal cancer

**DOI:** 10.1186/1471-2407-13-439

**Published:** 2013-09-27

**Authors:** Vlad Popovici, Eva Budinska, Fred T Bosman, Sabine Tejpar, Arnaud D Roth, Mauro Delorenzi

**Affiliations:** 1 Institute of Biostatistics and Analyses, Masaryk University, Kotlarska 2, Brno, 611 37, Czech Republic; 2 Bioinformatics Core Facility, Swiss Institute of Bioinformatics, Lausanne, Switzerland; 3 Institute of Pathology, Lausanne University Medical Center, Lausanne, Switzerland; 4 University Hospital Gasthuisberg, Katholieke Universiteit Leuven, Leuven, Belgium; 5 Oncosurgery Unit, Geneva University Hospital, Geneva, Switzerland; 6 University of Lausanne, Lausanne, Switzerland

**Keywords:** Colorectal cancer, BRAF V600E mutation, KRAS mutations, Survival analysis, Stratified analysis

## Abstract

**Background:**

The mutation status of the BRAF and KRAS genes has been proposed as prognostic biomarker in colorectal cancer. Of them, only the BRAF V600E mutation has been validated independently as prognostic for overall survival and survival after relapse, while the prognostic value of KRAS mutation is still unclear. We investigated the prognostic value of BRAF and KRAS mutations in various contexts defined by stratifications of the patient population.

**Methods:**

We retrospectively analyzed a cohort of patients with stage II and III colorectal cancer from the PETACC-3 clinical trial (N = 1,423), by assessing the prognostic value of the BRAF and KRAS mutations in subpopulations defined by all possible combinations of the following clinico-pathological variables: T stage, N stage, tumor site, tumor grade and microsatellite instability status. In each such subpopulation, the prognostic value was assessed by log rank test for three endpoints: overall survival, relapse-free survival, and survival after relapse. The significance level was set to 0.01 for Bonferroni-adjusted p-values, and a second threshold for a trend towards statistical significance was set at 0.05 for unadjusted p-values. The significance of the interactions was tested by Wald test, with significance level of 0.05.

**Results:**

In stage II-III colorectal cancer, BRAF mutation was confirmed a marker of poor survival only in subpopulations involving microsatellite stable and left-sided tumors, with higher effects than in the whole population. There was no evidence for prognostic value in microsatellite instable or right-sided tumor groups. We found that BRAF was also prognostic for relapse-free survival in some subpopulations. We found no evidence that KRAS mutations had prognostic value, although a trend was observed in some stratifications. We also show evidence of heterogeneity in survival of patients with BRAF V600E mutation.

**Conclusions:**

The BRAF mutation represents an additional risk factor only in some subpopulations of colorectal cancers, in others having limited prognostic value. However, in the subpopulations where it is prognostic, it represents a marker of much higher risk than previously considered. KRAS mutation status does not seem to represent a strong prognostic variable.

## Background

Our current models of colorectal cancer (CRC) are dominated by the idea of a sequential tumor progression from adenoma to carcinoma, in which the accumulation of genetic events in key genes defines alternative oncogenic paths with impact on tumor characteristics. These genetic events include the mutational activation of oncogenes like BRAF and KRAS, disruption of WNT signaling, allelic imbalance on chromosome 18q and mutation of TP53 tumor suppressor gene [1-4]. Since the mutations of BRAF and KRAS genes, which lead to the activation of MEK/ERK pathway, are seen as important events in the tumor progression and based on their relatively high incidence (7-15% for BRAF mutations and 35-40% for KRAS mutations [5-8]), they have been proposed as prognostic biomarkers for CRC. Of them, only BRAF V600E mutation has been consistently validated, while the prognostic value of KRAS mutation remains debatable. The BRAF has been shown to be prognostic for overall survival (OS) and survival after relapse (SAR) in general CRC population by us and others [9-13] as well as in microsatellite-stable (MSS) population [12,14], while having no prognostic value for relapse-free survival (RFS). In these studies, the hazard ratios (HR) for BRAF mutation varied between 1.4 and 2.1 for OS and 2.3 to 3.6 for SAR. In the case of KRAS mutation, the published results are contradictory, with prognostic value, in the positive studies, found only for relapse-free survival [9,11,15], while other studies, including our own [13], did not find any evidence of prognostic value for KRAS mutation. Also, a recent meta-analytical review found no evidence supporting the prognostic value of KRAS mutation [16]. A detailed review is given in [17].

The question remains whether the prognostic value of the BRAF and KRAS mutations is uniform across different patient groups defined by clinical parameters or if there are interactions that would influence their utility. Taking advantage of a large series of stage II-III CRC tumors with mutation data from the PETACC-3 clinical trial [18], we systematically investigate the prognostic value of the BRAF and KRAS mutations in all possible stratifications – contexts – defined by a set of clinical parameters found to be important in survival prognosis in a previous analysis [19]. The main question our study tries to answer is whether the mutations of BRAF and KRAS genes are indicators of different prognosis within otherwise uniform (with respect to the clinical parameters considered) subpopulations of patients with CRC. A secondary question we address, for the main findings, is whether the observed prognostic values are statistically significant also in multivariate models, in the respective subpopulations.

## Methods

We retrospectively analyzed the PETACC-3 clinical trial [18] data set (N = 1,423), of patients with stage II and III CRC, by generating the subpopulations defined by all possible combinations of levels of the following five variables: MSI status (MSI-H and MSS levels), tumor site (left and right), T stage (T1,2, T3, and T4), N stage (N0, N1 and N2) and tumor grade (G1,2 and G3,4). In total, there were 393 possible subpopulations (see Additional file 1 for an exhaustive listing), of which only those with more than N = 20 samples were further considered for testing the prognostic value of the BRAF and KRAS mutations. The full description of the data set is given in [19].

In each subpopulation, the prognostic importance of the BRAF and KRAS mutations was assessed using log-rank test comparing the survival of BRAF-/KRAS-mutant population to the BRAF- and KRAS- wild type (double wild type – WT2) population, for overall survival (OS), relapse-free survival (RFS) and survival after relapse (SAR) endpoints. Data was summarized with hazard ratios (HR), their 95% confidence intervals (CI), P-values and adjusted P-values (Bonferonni correction, denoted hereinafter by P^*^). For a result to be considered statistically significant we required that P^*^ ≤ 0.01 and that at least 10 patients were in each of the two groups compared. If only P ≤ 0.05, the result was reported as a trend towards significance. The significance of the interactions was tested by Wald test in the presence of both main effects, with significance level of 0.05 (no adjustment for multiple testing in this case). All tests were two-sided.

All computations were carried out in R version 2.15.2 (http://www.r-project.org) and survival analysis was performed using R survival package version 2.37-2.

## Results and discussion

In the global population, the BRAF mutation is prognostic for poorer overall survival and survival after relapse, while KRAS mutation is not prognostic for any of the three endpoints (Table 1). In stratified analyses and after correction for multiple testing, BRAF mutation status remained a significant prognostic marker in various subpopulations. On the contrary, KRAS mutation status never reached the level of significance required after P-value adjustment (P^*^ ≤ 0.01 and at least 10 patients in both of the groups compared). However, in several stratifications, KRAS mutation showed a trend towards significance (P ≤ 0.05). The full table of results with all possible stratifications is given as Additional file 1.

**Table 1:** Univariate analysis of the prognostic factors in the whole CRC population

		**OS**		**RFS**		**SAR**	
**Factor**	**Comparison**	**P-value**	**HR (95% CI)**	**P-value**	**HR (95% CI)**	**P-value**	**HR (95% CI)**
MSI	MSI-H vs MSS	0.0002	0.45 (0.30,0.69)	< 0.0001	0.48 (0.34,0.68)	0.9643	0.99 (0.65,1.52)
Site	Left vs Right	0.3143	0.89 (0.72,1.11)	0.2123	1.13 (0.93,1.36)	<0.0001	0.59 (0.47, 0.73)
Grade	G3,4 vs G1,2	0.0018	1.63 (1.29,2.23)	0.0012	1.56 (1.19,2.04)	0.0387	1.38 (1.01,1.88)
T stage	T3 vs T1,2	0.0634	1.76 (0.96,3.22)	0.0629	1.58 (0.97,2.58)	0.1399	1.57 (0.86,2.88)
	T4 vs T1,2	0.0002	3.06 (1.63,5.74)	< 0.0001	2.69 (1.61,4.48)	0.0680	1.78 (0.95,3.35)
N stage	N1 vs N0	< 0.0001	1.91 (1.38,2.65)	< 0.0001	1.78 (1.36, 2.32)	0.9809	0.98 (0.71,1.35)
	N2 vs N0	< 0.0001	4.51 (3.28,6.21)	< 0.0001	4.06 (3.11,5.29)	0.1498	1.24 (0.90,1.71)
BRAF	BRAF mut vs WT2	0.0004	1.92 (1.33,2.78)	0.0832	1.35 (0.96,1.89)	< 0.0001	2.56 (1.75,3.70)
	BRAF mut vs BRAF wt	0.0009	1.78 (1.26,2.53)	0.1174	1.30 (0.94,1.81)	< 0.0001	2.48 (1.74,3.53)
KRAS	KRAS mut vs WT2	0.1461	1.20 (0.93,1.54)	0.4410	1.09 (0.88,1.33)	0.1755	1.18 (0.93,1.52)
	KRAS mut vs KRAS wt	0.4826	1.09 (0.86,1.37)	0.7245	1.04 (0.85,1.27)	0.7222	1.04 (0.82,1.32)

### BRAF mutation

The BRAF mutation was prognostic for overall survival in MSS and/or left-sided tumors subpopulations (Figure 1). In the MSS tumors, BRAF was indicative of worse overall survival (P^*^ < 0.0001; HR = 2.82; 95% CI = 1.85 to 4.30), as well as in MSS/left tumors (P^*^ < 0.0001; HR = 6.41; 95% CI = 3.57 to 11.52) and all left-sided tumors (P^*^ < 0.0001; HR = 5.18; 95% CI = 3.00 to 8.94) (Figure 1A,B). At the same time, BRAF mutation was not prognostic in any stratification involving only right-sided tumors (Figure 1C) and/or MSI-H tumors. In a multivariate model, including up to second degree interactions between MSI status, BRAF mutation and tumor site, adjusted for grade, T stage and N stage, the only significant interaction was between BRAF mutation and tumor site (P = 0.0041). The interaction between BRAF mutation status and tumor site was also significant within MSS tumors (P = 0.0033), but not within MSI-H tumors. The interaction between BRAF mutation status and MSI status was not significant in either left or right-sided tumors. These results show that BRAF mutation represents an additional risk factor only within MSS/left tumors, with no statistically significant effect in right or MSI-H tumors, the general prognostic value of BRAF mutation being driven by its effect in this subpopulation. As a consequence, the corresponding HR should be re-interpreted: a BRAF mutation does not double the risk of death for all patients carrying this mutation (HR = 1.92 in global population), but represents a six-fold increase of the risk in the case of patients with MSS/left tumors (HR = 6.41) – in comparison with the double wild type MSS/left tumors. At the same time, BRAF mutation does not significantly influence the risk of death (in comparison with WT2) in MSI-H and/or right-sided tumors. The MSS/left side BRAF-mutant population emerges as the worst surviving group of patients in our data set: for example, the 3-year overall survival rate is 0.35 (95% CI = 0.20 to 0.66) in comparison to 0.89 (95% CI = 0.85 to 0.93) for KRAS-mutant and 0.91 (95% CI = 0.88 to 0.93) for WT2, respectively (Table 2). The observation could not be extended to MSS/right-sided tumors (Table 2).

**Figure 1:** **Overall survival: prognostic value of BRAF and KRAS mutations within MSS and by tumor site. A**: all MSS tumors; **B**: MSS left-sided tumors; **C**: MSS right-sided tumors. The light gray survival curve represents the whole subpopulation survival (**A**: all MSS, **B**: MSS left-sided, **C**: MSS right-sided tumors).

**Table 2:** Three-year overall and relapse-free survival rates, and one-year survival after relapse rates in MSS/left and MSS/right populations, stratified by mutation status

	**MSS/left**		**MSS/right**	
**Population**	**Survival rate**	**95% CI**	**Survival rate**	**95% CI**
OS: 3-year survival rates				
WT2	0.91	0.88-0.93	0.83	0.77-0.89
KRAS mut	0.89	0.85-0.93	0.80	0.74-0.86
BRAF mut	0.37	0.20-0.66	0.73	0.60-0.89
RFS: 3-year survival rates				
WT2	0.75	0.71-0.80	0.75	0.68-0.82
KRAS mut	0.68	0.62-0.74	0.73	0.66-0.80
BRAF mut	0.32	0.16-0.61	0.68	0.54-0.84
SAR: 1-year survival rates				
WT2	0.81	0.74-0.88	0.65	0.52-0.82
KRAS mut	0.80	0.71-0.89	0.75	0.53-0.80
BRAF mut	0.17	0.05-0.60	0.36	0.17-0.79

Interestingly, BRAF mutation was also prognostic for shorter relapse-free survival in left-sided tumors (Figure 2): all left-sided tumors (P^*^ = 0.0002; HR = 3.31; 95% CI = 1.98 to 5.55) and MSS/left tumors (P^*^ = 0.0005; HR = 3.57; 95% CI = 2.02 to 6.31) (Figure 2, see also Table 2). This is a novel observation, since BRAF mutation was not generally considered prognostic for relapse. In other MSS-subpopulations involving left-sided tumors BRAF mutation is also prognostic (see Additional file 1). Again, the BRAF mutation was not prognostic in any subpopulation involving MSI-H and/or right-sided tumors. In a multivariate model, involving up to second degree interactions between MSI status, BRAF mutation and tumor site, adjusted for grade, T stage and N stage, the only significant interaction was between BRAF mutation and tumor site (P = 0.047). The interaction between BRAF mutation status and tumor site was also significant within MSS tumors (P = 0.043), but not within MSI-H tumors (where the small number of BRAF mutants in the left colon limits the statistical power). Hence, the prognostic value of the BRAF mutation is confined to the MSS/left-sided tumors.

**Figure 2:** **Relapse-free survival: prognostic value of BRAF and KRAS in left-sided tumors. A**: all left-sided tumors; **B**: MSS left-sided tumors. The light gray survival curve represents the whole subpopulation survival (**A**: all left tumors; **B**: MSS left).

For the survival after relapse (SAR), BRAF mutation represents an additional risk factor in more stratifications, most of them involving MSS and/or left-sided tumors. BRAF mutation shows also a trend to be prognostic in MSS/right-sided tumors as well, even though the p-value was no longer significant after multiple testing correction. The BRAF mutation was indicative of poor survival after relapse in all MSS tumors (P^*^ < 0.0001; HR = 3.43; 95% CI = 2.19 to 5.36); MSS/left tumors (P^*^ = 0.0002; HR = 3.89; 95% CI = 2.11 to 7.20) and showed a trend in MSS/right (P = 0.0111; HR = 2.27; 95% CI = 1.17 to 4.38) (Figure 3). The test for interaction between BRAF mutation status and tumor site was not significant, hence we conclude that BRAF mutation is prognostic for SAR in all MSS patients.

**Figure 3:** **Survival after relapse: prognostic value of BRAF and KRAS mutations in MSS tumors by site. A**: all MSS tumors; **B**: MSS left-sided tumors; **C**: MSS right-sided tumors. The light gray survival curve represents the whole subpopulation survival (**A**: all MSS, **B**: MSS left-sided, **C**: MSS right-sided tumors).

The differences in prognostic value of the BRAF mutation status in various subpopulations suggest a certain degree of heterogeneity in the survival of patients harboring this mutation. Indeed, within the BRAF mutant population, the MSS tumors had worse outcome for overall survival (P = 0.0021; HR = 3.45; 95% CI = 1.49 to 7.69)) and relapse-free survival (P = 0.0085; HR = 2.63; 95% CI = 1.25 to 5.56), this observation being in line with the fact that MSI-H has a protective prognostic effect in CRC. At the same time, the left BRAF-mutant tumors had a worse prognosis than the right BRAF-mutant tumors, for overall survival (within all BRAF-mutants: P = 0.0003; HR = 3.20; 95% CI = 1.64 to 6.23; within MSS/BRAF-mutants: P = 0.0059; HR = 2.84; 95% CI = 1.31 to 6.15; while within MSI-H/BRAF-mutants it could not be assessed) and for relapse-free survival (within all BRAF-mutants: P = 0.0002; HR = 3.24; 95% CI = 1.71 to 6.16; within MSS/BRAF-mutants: P = 0.0062; HR = 2.82; 95% CI = 1.30 to 6.12; while within MSI-H/BRAF-mutants it could not be assessed). However, there was no statistically significant difference in survival after relapse among BRAF mutants, all having an equally poor survival.

### KRAS mutation

KRAS mutation did not reach the significance level required to be considered prognostic for any of the three endpoints, since the adjusted p-values were all larger than 0.01. However, in some cases, it showed a trend towards significance (P ≤ 0.05).

In overall survival, KRAS mutation had a trend to become significant in several stratifications of tumors with early stage lymph node invasion (N1). In all these, KRAS mutation was a marker of worse outcome (see Additional file 1). While not being a significant prognostic factor (as required by us) for relapse-free survival, KRAS mutation showed a trend to become prognostic. In contrast with BRAF, KRAS mutation seemed to be prognostic for RFS mostly in the right colon. The most intriguing observation was in MSI-H/right colon subpopulation (N = 102, KRAS mutants: 39), where KRAS mutation seemed to identify a low risk group (P = 0.0349; HR = 0.29; 95% CI = 0.08 to 0.99) (Figure 4). KRAS mutation was not prognostic for SAR. Also, no significant interaction between KRAS mutation, MSI status and tumor site was observed, for any of the three endpoints.

**Figure 4:** **Relapse-free survival: prognostic value of BRAF and KRAS in MSI-H tumors by site. A**: all MSI-H tumors; **B**: MSI-H left-sided tumors; **C**: MSI-H right-sided tumors. The light gray survival curve represents the whole subpopulation survival (**A**: all MSI-H, **B**: MSI-H left-sided, **C**: MSI-H right-sided tumors).

Since several studies have suggested that KRAS mutations at codon 12 may have a different prognostic value than codon 13 mutations [20], we have tested for differences in survival between the two groups of mutations, in all the same stratifications. No statistically significant difference was observed, but the sample size of our data might be too limited to detect such differences.

## Conclusions

In our analyses, we have compared the survival of BRAF/KRAS-mutated population with that of the double-wild type population, while controlling for several other parameters (tumor site, T and N stage, grade and MSI status).

Our analyses confirm the prognostic value of BRAF mutation status, in various stratifications. As a novelty, we observe a strong prognostic value for relapse-free survival of the BRAF mutation status in the MSS/left-colon tumors.

The interpretation of BRAF mutation as additional risk factor has to be made in the context of MSI status and tumor location. Indeed, our results show that BRAF represents a risk factor in the left colon and/or MSS tumors. In the data analyzed, we found no sufficient statistical evidence supporting a worse outcome associated with BRAF mutation in MSI-H tumors. As a consequence, the published hazard ratios for BRAF mutation for general population have to be reconsidered. The tumor staging (T or N stage, tumor grade) had a lesser impact on the prognostic value of the BRAF mutation status, while the tumor background (site and microsatellite (in)stability) significantly influenced the prognostic.

For the KRAS mutation, we could not confirm nor completely disprove its prognostic value. It was prognostic in several stratifications, in some showing a protective effect, while in others representing a risk factor. This is probably an effect of the heterogeneity of KRAS mutant population [21,22] and may explain in part the contradictory results published so far. With the strict requirements for statistical significance imposed, KRAS mutation did not appear to have prognostic value in any of the stratifications. The trend towards significance suggests, however, a potential utility as prognostic marker for RFS mostly in right colon.

In conclusion, the utility of the BRAF and KRAS as prognostic biomarkers depends on the MSI status and tumor location. We hypothesize that this interaction may extend to other biomarkers and prognostic gene signatures as well. At the same time, this observation has clear implications in clinical trial design and needs to be accounted for.

We make public the full table with all stratifications to support similar analyses in other data sets.

## Abbreviations

MSI: Microsatellite instability; MSI-H: High microsatellite instability; MSS: Microsatellite stable; OS: Overall survival; RFS: Relapse-free survival; SAR: Survival after relapse; WT2: Double wild type tumors: tumors that are BRAF- and KRAS-wild type.

## Competing interests

The authors declare that they have no competing interests.

## Authors’ contributions

VP conceived and designed the investigation, performed the statistical analyses, interpreted the results and drafted the manuscript. EB performed statistical analyses and drafted the manuscript. FB, ST, AR and MD participated in data generation, result interpretation and contributed to manuscript drafting. All authors have read and approved the final manuscript.

## Pre-publication history

The pre-publication history for this paper can be accessed here:

http://www.biomedcentral.com/1471-2407/13/439/prepub

## Supplementary Material

Additional file 1 **Full survival analysis results.** In each possible stratification three endpoints were tested - overall survival, relapse-free survival and survival after relapse - and the sample size of the analysis along with the resulting p-values and hazard ratios are given. Click here for file
